The article "Diagnostic Value of Prostate-Specific Antigen Combined with Plasma miRNA-149 Expression in Patients with Prostate Cancer Based on Experimental Data and Bioinformatics" was published in 2022. Journal: Contrast Media Mol Imaging.

# Diagnostic Value of Prostate-Specific Antigen Combined with Plasma miRNA-149 Expression in Patients with Prostate Cancer Based on Experimental Data and Bioinformatics

**DOI:** 10.1155/2022/6094409

**Published:** 2022-07-22

**Authors:** Hao Wang, Ling Yang, Ying Mi, Yanan Wang, Chunmei Ma, Jing Zhao, Ping Liu, Yu Gao, Peijun Li

**Affiliations:** Department of Urology, General Hospital of Ningxia Medical University, Yinchuan, Ningxia Hui Autonomous Region, China

## Abstract

**Purpose:**

The aim of this study is to explore the diagnostic value of prostate-specific antigen (PSA) combined with serum miRNA-149 expression in prostate cancer (PCa) by conducting experiments and bioinformatics analysis. *Patients and Methods*. 50 PCa patients were enrolled on the experimental group from January 2020 to December 2021. 56 patients with benign prostatic hyperplasia (BPH) were selected as the control group at the same time. Real-time fluorescent quantitative PCR was applied to investigate the miRNA-149 expression. PSA was detected by using a chemiluminescence meter using Abbott i4000. Applying bioinformatics analysis, we explored the expression of hsa-miR-149 in PCa in The Cancer Genome Atlas (TCGA) database. Kaplan–Meier analyses were used to evaluate the prognostic value, and the ROC curve was applied.

**Results:**

The expression level of miRNA-149 in the PCa group was significantly higher than that in the BPH group (*P* < 0.05). The PSA level in the PCa group was also significantly higher than that in the BPH group (*P* < 0.05). TCGA data analysis revealed that PCa tissues had significantly increased hsa-miR-149 expression. The results of survival analysis showed that patients with high expression of hsa-miR-149 had better prognosis. Additionally, the pathological N stage of PCa correlates with the hsa-miR-149 expression level (*P* = 0.002). According to ROC curve analysis, the region under the curve was 0.653, 95% CI: 0.576–0.730.

**Conclusion:**

High expression of serum miRNA-149 is associated with PCa patients. Although combined PSA did not improve the diagnostic efficacy, miRNA-149 has high specificity in the diagnosis of PCa. miRNA-149 might be a novel marker for early diagnosis and prognosis assessment for PCa.

## 1. Introduction

Prostate cancer (PCa) is a common malignant tumor in men, with a relatively low incidence in China, but a high incidence in Europe, United States, and other developed areas [1]. Among the malignant tumors that have great harm to men's health, PCa ranks the second. PCa does not show a high overall incidence in China. According to the data from the national tumor registry in 2015, prostate cancer ranked 6th in the incidence of male malignant tumors, accounting for 3.35% of the incidence of male malignant tumors [2]. It ranks 10th in male malignant tumor mortality, accounting for 2.1% of male malignant tumor deaths [2]. In the national tumor registration area, prostate cancer ranks first in the incidence of male genitourinary malignancy in China, higher than bladder cancer [3]. However, morbidity is increasing in recent years. The patients usually do not show obvious symptoms in the early stage. Some patients are prone to lower urinary tract syndrome and other clinical symptoms. Nevertheless, they are generally caused by concurrent diseases such as prostate hyperplasia. With further development, the symptoms continue to worsen. When bone metastasis occurs in some patients, the pain of metastatic lesions in the pelvic area, waist or pathological fracture may be the main clinical manifestations. The early stage of PCa has no typical symptoms, resulting in about 20% of patients having metastases when diagnosed and missing the optimal surgical treatment period. Therefore, the research on PCa focuses on early diagnosis. Currently, the most commonly used screening and early diagnosis of PCa includes a combination of digital rectal examination (DRE) and prostate-specific antigen (PSA). In recent years, PSA has played an important role in PCa screening. However, as the most widely used diagnostic marker, PSA has high sensitivity but low specificity [4, 5]. Therefore, finding one biomarker with high sensitivity and specificity for early diagnosis has become the hope of medical personnel and researchers. Furthermore, with the introduction of “liquid biopsy,” more and more relevant laboratory indicators have received clinical attention [6]. In recent years, related study confirms that the miRNAs play a key role; especially in the development of tumor has been shown to play an important role in the process, have certain specificity, and can be used as an index of early diagnosis. It was reported that miRNA-149 promoted tumor growth and metastasis and acts as “oncogene” [7, 8]. Based on experiment and bioinformatics analysis, the present study investigated the miRNA-149 expression and the diagnostic efficacy of miRNA-149 alone and combined with PSA in PCa.

The article "Diagnostic Value of Prostate-Specific Antigen Combined with Plasma miRNA-149 Expression in Patients with Prostate Cancer Based on Experimental Data and Bioinformatics" was published in 2022. Journal: Contrast Media Mol Imaging.

## 2. Materials and Methods

### 2.1. Patients and Controls

A total of 50 PCa patients were enrolled in the experimental group from January 2018 to December 2021, and all cases were confirmed by histopathology. During the same period, 56 patients with benign prostatic hyperplasia (BPH) were enrolled in the control group. Patients with cardiac and renal failure, severe hepatobiliary diseases, and other malignant tumors were excluded. There was no significant difference in age or sex among the two groups (*P* > 0.05). The present study was examined and approved by the Ethics Committee of the General Hospital of Ningxia Medical University. PCa patients and BPH patients directly signed the informed consent. The current research complies with the Declaration of Helsinki.

### 2.2. RNA Extraction

2 ml fasting venous blood was collected in the morning for the observation group and control group. All blood samples were centrifuged at 2000 r/min for 15 min with an effective centrifugation radius of 6 cm. Serum samples were gathered and kept in a refrigerator at −70°C. Repeated freeze-thaw and hemolysis were avoided in all specimens. 300 *μ*L of serum was taken from patients, and total RNA was extracted using the mirVanaTPAISTM miRNA kit (Applied Biosystems). miRNA was isolated and extracted according to the ABI miRNA extraction kit (Applied Biosystems), and reverse transcription was performed strictly according to kit instructions.

### 2.3. Real-Time Fluorescence Quantitative PCR (qRT-PCR)

Total TaqMan MicroRNA Reverse was applied with 5 *μ*L RNA as a template. Transcription was performed by using the Transcription kit (ABI), the total Transcription system is 15 *μ*L, and the reaction conditions are as follows: 16°C for 30 min, 42°C for 30 min, 85°C for 5 min, reverse transcription primer miRNA-149-specific stem-loop primer was performed for TaqMan MicroRNA Assay ABI, which upstream sequence 5′-AGCAGCAUUGUACAGGGCUAUCA-3′ and 3′-AUAGCCCUGUACAAUGCUGCUUU-5′ downstream; Upstream sequence of internal reference gene: 5′-UUCUCCGAACGUGUCACGUTT-3′, downstream sequence: 3′-ACGUGACACGUUCGGAGAATT-5′. The reverse transcription primers, PCR primers, and probes of miRNA-149 were obtained from ABI Bio TaqMan miRNA RT Kit and TaqMan miRNA Assay Kit. The total fluorescence quantitative PCR reaction system was 20 *μ*L, and reaction conditions were 95°C for 10 min, 95°C for 15 s, 60°C for 1 min, and 40 cycles. All the reactions were performed on ABI 7500 real-time quantitative PCR instrument, and each sample was repeated three times, with U6 as the reference gene. The 2^−△△Ct^ method was used to calculate miRNA-149 relative quantitative expression level (△Ct = Ct_miRNA-149_ − CT_U6_).

### 2.4. Bioinformatics Analysis

The miRNA expression profiles of prostate cancer samples and adjacent normal tissues were acquired from TCGA using the UCSC Xena Browser (https://xenabrowser.net/) [9–13]. The clinicopathological data of the patients with intact survival information, including age at initial pathologic diagnosis, histology, tumor grade, clinical stage, and living status, were downloaded for survival-related analysis.

The article "Diagnostic Value of Prostate-Specific Antigen Combined with Plasma miRNA-149 Expression in Patients with Prostate Cancer Based on Experimental Data and Bioinformatics" was published in 2022. Journal: Contrast Media Mol Imaging.

### 2.5. Statistical Analysis

The SPSS 17.0 statistical software was used for analysis. Measurement data were expressed as mean ± standard deviation (*X* ± *S*) between two groups. Two independent sample *T*-tests were used for comparison, and a single factor was used for comparison between multiple groups. ANOVA analysis and LSD-T test were performed. Statistical tests of bioinformatics analysis were conducted through R (version 4.0.3). Comparisons between two groups were performed via Wilcoxon rank-sum test. Kaplan–Meier curves for overall survival were generated, and the difference between groups was compared with the log-rank test.

## 3. Results

### 3.1. miRNA-149 Expression and PSA in Prostate Cancer and Benign Prostatic Hyperplasia

The relative expression levels of miRNA-149 in serum of PCa and BPH patients are shown in Figure 1. The expression level of miRNA-149 in the PCa group (15.19 ± 4.44) was significantly higher than that in the BPH group (9.35 ± 1.54), and the difference was statistically significant (*P* < 0.05). A similar result was also found in PSA, which was shown in Figure 2.

### 3.2. Diagnostic Efficacy of miRNA-149 Alone and in Combination with PSA

Compared with PSA, miRNA-149 had lower AUC, Yuden index, sensitivity, and higher specificity in the diagnosis of PCa. miRNA-149 combined with PSA did not improve the diagnostic efficacy of PCa, as shown in Table 1.

### 3.3. Bioinformatics Analysis

To determine whether hsa-miR-149 expression was a prognostic factor for poor survival, expression data from the TCGA dataset were analyzed. Accordingly, PCa tissues had a higher hsa-miR-149 expression level than normal prostate tissues (Figure 3) and Kaplan–Meier analysis showed that low hsa-miR-149 expression was associated with poor prognosis (Figure 4). Furthermore, we explored the relationship between hsa-miR-149 expression level and clinicopathological characteristics. Our results showed that the level of hsa-miR-149 expression only increased significantly in the pathological N stage (Figure 5). The ROC analysis was performed for hsa-miR-149 in the TCGA dataset, which showed the robust capacity of predictive performance: AUC = 0.653, (95% CI: 0.576–0.730) (Figure 6). These findings suggested that hsa-miR-149 may play a crucial role in PCa development.

## 4. Discussion

There are regional differences in the incidence of PCa, and its incidence in areas with high incidence is about 20 times higher than that in areas with low incidence [14]. As the early symptoms of PCa are not typical, there are many clinical symptoms similar to prostate hyperplasia. The main screening methods include PSA and DRE. Diagnosis depends on the color ultrasound-guided needle biopsy of the prostate. PSA is an important tumor marker for the diagnosis and prognosis of PCa, but as an indicator of early screening of prostate cancer, PSA is not sensitive and specific enough. Therefore, it is urgent to find a more accurate tumor marker to achieve the goal of early diagnosis and treatment of prostate cancer.

The article "Diagnostic Value of Prostate-Specific Antigen Combined with Plasma miRNA-149 Expression in Patients with Prostate Cancer Based on Experimental Data and Bioinformatics" was published in 2022. Journal: Contrast Media Mol Imaging.

Exosomes were first discovered by Trams et al. in 1980. With a straight diameter of 30–100 nm, exosomes contain a variety of proteins, DNA, mRNA, and miRNA. They are vesicles formed by cell membrane fusion and efflux in the process of cell entosis and are widely found in body fluids, such as serum, saliva, and urine. Exosomes are abundant in tumor microenvironment, which is closely related to the occurrence and development of tumor, immune escape, and the establishment of the microenvironment. Studies have shown that exosomes derived from tumor cells can be used for the early detection of tumors. miRNAs in exosomes are a class of noncoding, 18–25 nt single-stranded small RNAs, which are involved in important physiological and pathological changes of cells, and abnormal expression of miRNAs has been observed in many tumors in studies [15–33].

Lawrie et al. were the first to confirm the presence of tumor-specific miRNA in serum, and they found the higher expression level of miRNA-21 in diffuse large B-cell lymphoma, and the expression level of miRNA-21 was correlated with the survival rate [34]. Chen et al. recently found that the expression profile of plasma microRNA can be used as a noninvasive marker of PCa [35]. Moreover, five miRNAs (LET-7C, LET-7E, miRNA-30C, miRNA-622, and miRNA-1285) could accurately distinguish PCa from BPH (AUC = 0.924) [35].

The present study investigated the potential role of hsa-miR-149 in prostate cancer. Analysis of the TCGA database revealed that hsa-miR-149 expression was upregulated in prostate cancer and that low hsa-miR-149 expression levels were positively correlated with poor survival. Moreover, our results showed that hsa-miR-149 expression levels were associated with the pathological N stage.

In this study, the relative expression of miRNA-149 in PCa and BPH serum was detected by qRT-PCR. It was found that miRNA-149 was highly expressed in PCa and could distinguish PCa and BPH with an AUC of 0.806, which was consistent with the results of Bryant et al. The AUC of PSA combined with miRNA-149 in distinguishing PCa from BPH was 0.96, and both sensitivity and specificity were 91%. As far as we know, this is the first study which investigates serum miRNA-149 expression in PCa. In recent years, circulating miRNA has been found not only as a marker for tumor diagnosis and prognosis but also as a potential method for personalized therapy [36]. Transrectal ultrasound-guided needle biopsy is the gold standard for PCa diagnosis in China. With the wide application of PSA in clinical practice, PCa diagnosis and treatment techniques are constantly improved, and PCa comprehensive treatment is becoming mature. With China entering an aging society, increasing life expectancy, living habits, and diet structure change, PCa incidence is rising and PCa patients diagnosed are late which leads to poorer prognosis and high mortality rate. Therefore, early screening of PCa should be advocated for middle-aged and elderly men. Because of simple laboratory conditions and limited funds, we have to admit the fact that the sample size of the current study is small. In future studies, we will include more patients and healthy people to make our results more reliable.

The article "Diagnostic Value of Prostate-Specific Antigen Combined with Plasma miRNA-149 Expression in Patients with Prostate Cancer Based on Experimental Data and Bioinformatics" was published in 2022. Journal: Contrast Media Mol Imaging.

## 5. Conclusion

High expression of serum miRNA-149 is associated with PCa patients. Although combined PSA did not improve the diagnostic efficacy, miRNA-149 has high specificity in the diagnosis of PCa. miRNA-149 might be a novel marker for early diagnosis and prognosis assessment for PCa.

## Figures and Tables

**Figure 1:** Expression level of miRNA-149 in both PCa group and BPH group. BPH, benign prostatic hyperplasia; PCa, prostate cancer.

**Figure 2:** Expression level of PSA in both PCa group and BPH group. BPH, benign prostatic hyperplasia; PSA, prostate-specific antigen; PCa, prostate cancer.

**Figure 3:** The relative expression of hsa-miR-149 in the TCGA dataset.

**Figure 4:** Kaplan–Meier analysis of overall survival according to high or low hsa-miR-149 expression in the TCGA database.

**Figure 5:** The relative expression of hsa-miR-149 across different pathological stages.

**Figure 6:** The ROC curve of hsa-miR-149 in the TCGA dataset.

**Table 1:** Diagnostic efficacy of miRNA-149 alone and in combination with PSA for PCa.

Indicators	AUC	Youden index	Sensitivity	Specificity
miRNA-149	0.71	0.32	0.33	0.98
PSA	0.96	0.82	0.91	0.91
Combination	0.96	0.82	0.91	0.91

PSA, prostate-specific antigen.

## Data Availability

All the data generated or analyzed during this study are included in this published article.

## References

[1] Litwin M. S., Tan H. J. (2017). The diagnosis and treatment of prostate cancer: a review. *JAMA*.

[2] Liu X., Yu C., Bi Y., Zhang Z. J. (2019). Trends and age-period-cohort effect on incidence and mortality of prostate cancer from 1990 to 2017 in China. *Public Health*.

[3] Fu Z. T., Guo X. L., Zhang S. W. (2020). [Statistical analysis of incidence and mortality of prostate cancer in China, 2015]. *Zhonghua Zhongliu Zazhi*.

The article "Diagnostic Value of Prostate-Specific Antigen Combined with Plasma miRNA-149 Expression in Patients with Prostate Cancer Based on Experimental Data and Bioinformatics" was published in 2022. Journal: Contrast Media Mol Imaging.

[4] Terada N., Akamatsu S., Kobayashi T., Inoue T., Ogawa O., Antonarakis E. S. (2017). Prognostic and predictive biomarkers in prostate cancer: latest evidence and clinical implications. *Ther Adv Med Oncol*.

[5] Chen R., Sjoberg D. D., Huang Y. (2017). Prostate specific antigen and prostate cancer in Chinese men undergoing initial prostate biopsies compared with western cohorts. *The Journal of Urology*.

[6] Hegemann M., Stenzl A., Bedke J., Chi K. N., Black P. C., Todenhofer T. (2016). Liquid biopsy: ready to guide therapy in advanced prostate cancer?. *BJU International*.

[7] Chen Y., Zhao J., Luo Y., Wang Y., Jiang Y. (2016). Downregulated expression of miRNA-149 promotes apoptosis in side population cells sorted from the TSU prostate cancer cell line. *Oncology Reports*.

[8] Luo Z., Zhang L., Li Z. (2012). An in silico analysis of dynamic changes in microRNA expression profiles in stepwise development of nasopharyngeal carcinoma. *BMC Medical Genomics*.

[9] Qiu Y., Li H., Xie J., Qiao X., Wu J. (2021). Identification of ABCC5 among ATP-binding cassette transporter family as a new biomarker for hepatocellular carcinoma based on bioinformatics analysis. *International Journal of General Medicine*.

[10] Xie J., Li H., Chen L. (2021). A novel pyroptosis-related lncRNA signature for predicting the prognosis of skin cutaneous melanoma. *International Journal of General Medicine*.

[11] Qiu Y., Li H., Zhang Q., Qiao X., Wu J. (2022). Ferroptosis-related long noncoding RNAs as prognostic marker for colon adenocarcinoma. *Applied Bionics and Biomechanics*.

[12] Xie J., Chen L., Sun Q. (2022). An immune subtype-related prognostic signature of hepatocellular carcinoma based on single-cell sequencing analysis. *Aging (Albany NY)*.

[13] Li C., Qu L., Matz A. J. (2022). AtheroSpectrum reveals novel macrophage foam cell gene signatures associated with atherosclerotic cardiovascular disease risk. *Circulation*.

[14] Coleman M. P., Quaresma M., Berrino F. (2008). Cancer survival in five continents: a worldwide population-based study (CONCORD). *The Lancet Oncology*.

[15] Lee Y. S., Dutta A. (2009). MicroRNAs in cancer. *Annual Review of Pathology: Mechanisms of Disease*.

[16] Di Leva G., Garofalo M., Croce C. M. (2014). MicroRNAs in cancer. *Annual Review of Pathology: Mechanisms of Disease*.

[17] Sun L., Jiang R., Li J. (2017). MicoRNA-425-5p is a potential prognostic biomarker for cervical cancer. *Annals of Clinical Biochemistry*.

[18] Park S., Eom K., Kim J. (2017). MiR-9, miR-21, and miR-155 as potential biomarkers for HPV positive and negative cervical cancer. *BMC Cancer*.

[19] Li M., Li B. Y., Xia H., Jiang L. L. (2017). Expression of microRNA-142-3p in cervical cancer and its correlation with prognosis. *European Review for Medical and Pharmacological Sciences*.

The article "Diagnostic Value of Prostate-Specific Antigen Combined with Plasma miRNA-149 Expression in Patients with Prostate Cancer Based on Experimental Data and Bioinformatics" was published in 2022. Journal: Contrast Media Mol Imaging.

[20] Angius A., Pira G., Scanu A. M. (2019). MicroRNA-425-5p expression affects BRAF/RAS/MAPK pathways in colorectal cancers. *International Journal of Medical Sciences*.

[21] Feng R., Chen X., Yu Y. (2010). miR-126 functions as a tumour suppressor in human gastric cancer. *Cancer Letters*.

[22] Li X., Zhang Y., Zhang H. (2011). miRNA-223 promotes gastric cancer invasion and metastasis by targeting tumor suppressor EPB41L3. *Molecular Cancer Research*.

[23] Wu Q., Jin H., Yang Z. (2010). MiR-150 promotes gastric cancer proliferation by negatively regulating the pro-apoptotic gene EGR2. *Biochemical and Biophysical Research Communications*.

[24] Lai K. W., Koh K. X., Loh M. (2010). MicroRNA-130b regulates the tumour suppressor RUNX3 in gastric cancer. *European Journal of Cancer*.

[25] Li X., Zhang Y., Shi Y. (2011). MicroRNA-107, an oncogene microRNA that regulates tumour invasion and metastasis by targeting DICER1 in gastric cancer. *Journal of Cellular and Molecular Medicine*.

[26] Liu T., Tang H., Lang Y., Liu M., Li X. (2009). MicroRNA-27a functions as an oncogene in gastric adenocarcinoma by targeting prohibitin. *Cancer Letters*.

[27] Xiao B., Guo J., Miao Y. (2009). Detection of miR-106a in gastric carcinoma and its clinical significance. *Clinica Chimica Acta*.

[28] Takagi T., Iio A., Nakagawa Y., Naoe T., Tanigawa N., Akao Y. (2009). Decreased expression of microRNA-143 and -145 in human gastric cancers. *Oncology*.

[29] Wada R., Akiyama Y., Hashimoto Y., Fukamachi H., Yuasa Y. (2009). miR-212 is downregulated and suppresses methyl-CpG-binding protein MeCP2 in human gastric cancer. *International Journal of Cancer*.

[30] Gao C., Zhang Z., Liu W., Xiao S., Gu W., Lu H. (2010). Reduced microRNA-218 expression is associated with high nuclear factor kappa B activation in gastric cancer. *Cancer*.

[31] Qiao M., Ding J., Yan J., Li R., Jiao J., Sun Q. (2018). Circular RNA expression profile and analysis of their potential function in psoriasis. *Cellular Physiology and Biochemistry*.

[32] Jiang K., Xie L. F., Xiao T. Z., Qiu M. Y., Wang W. L. (2019). MiR-181d inhibits cell proliferation and metastasis through PI3K/AKT pathway in gastric cancer. *European Review for Medical and Pharmacological Sciences*.

[33] Luo X., Burwinkel B., Tao S., Brenner H. (2011). MicroRNA signatures: novel biomarker for colorectal cancer?. *Cancer Epidemiology, Biomarkers & Prevention*.

[34] Lawrie C. H., Gal S., Dunlop H. M. (2008). Detection of elevated levels of tumour-associated microRNAs in serum of patients with diffuse large B-cell lymphoma. *British Journal of Haematology*.

The article "Diagnostic Value of Prostate-Specific Antigen Combined with Plasma miRNA-149 Expression in Patients with Prostate Cancer Based on Experimental Data and Bioinformatics" was published in 2022. Journal: Contrast Media Mol Imaging.

[35] Chen Z. H., Zhang G. L., Li H. R. (2012). A panel of five circulating microRNAs as potential biomarkers for prostate cancer. *The Prostate*.

[36] Chandra V., Kim J. J., Mittal B., Rai R. (2016). MicroRNA aberrations: an emerging field for gallbladder cancer management. *World Journal of Gastroenterology*.

